# Clinical Significance of Hyperdense Lesions on Non-enhanced Brain CT Obtained Immediately after Arterial Revascularization in Acute Ischemic Stroke Patients

**DOI:** 10.1155/2021/1562502

**Published:** 2021-09-03

**Authors:** Changbin Wang, Zudong Yin, Xinyi Zhang, Xiumin Zhao

**Affiliations:** ^1^Department of Radiology, Shandong Provincial Third Hospital, Cheeloo College of Medicine, Shandong University, Jinan 250031, China; ^2^Department of Neurology, Shandong Provincial Third Hospital, Cheeloo College of Medicine, Shandong University, No. 12, Wuyingshan Middle Road, Tianqiao District, Jinan 250031, China

## Abstract

**Purpose:**

To analyze the characteristics of hyperdense lesions on brain CT conducted immediately after arterial revascularization (AR) in patients with acute ischemic stroke (AIS), track the outcome of those lesions and investigate their clinical significance.

**Materials and Methods:**

97 AIS patients were enrolled in our study. Among them, 52 patients showed hyperdense lesions and were divided into three categories: type I, type II and type III according to the morphologic characteristics of hyperdense lesions. All patients underwent several follow-up CT/MR examinations to visualize the outcomes of the lesions.

**Results:**

Among the 52 patients, 22 showed contrast extravasation, 23 displayed contrast extravasation combined with hemorrhagic transformation (HT) and 7 confirmed symptomatic intracranial hemorrhage (SICH) in follow-up CT/MR. Among the without hyperdense lesions group, only 7 converted to hemorrhage, and no SICH occurred. All type I lesions showed contrast extravasation; 23 type II lesions turned to hemorrhage, 2 revealed SICH and 6 were pure contrast extravasation; all of the type III developed into SICH.

**Conclusion:**

Hyperdense lesions on non-enhanced brain CT obtained immediately after arterial revascularization (AR) exhibited varying features. Type I indicated a pure contrast extravasation. Type II and type III hyperdense lesions suggested higher incidence of HT, the presence of type III lesions indicated an ominous outcome.

## 1. Introduction

Arterial revascularization (AR) has become the preferred treatment for patients with acute ischemic stroke (AIS) [1–3]. Non-enhanced brain CT conducted immediately after AR often presents hyperdense lesions in the parenchyma [4, 5]. Such hyperdense lesions have been reported and analyzed in various literature since 1993 [6]. However, it is still a tricky problem to determine whether the hyperdense lesions are contrast extravasation or cerebral hemorrhage [7]. The purpose of this study was to analyze the imaging characteristics of intracranial hyperdense lesions and to classify them according to their morphological characteristics. And the final outcome and clinical significance of different types of hyperdense lesions was analyzed based on its spontaneous regression, HT, or even SICH.

## 2. Materials and Methods

### 2.1. Patients

From August 2016 to Match 2020, 97 AIS patients (51 males and 46 females) were included in our study with an average age of 61.73 ± 8.44 years (range, 41-83 years). This study was approved by the Medical Ethics Committee of our hospital. Written informed consent was obtained from all patients.

### 2.2. Arterial Thrombolysis or/and Mechanical Thrombectomy

All patients received arterial thrombolysis or/and mechanical thrombectomy within 6 hours after onset. The findings of brain CT immediately after AR were analyzed in all cases. The contrast agent used for cerebral angiography during AR was iohexol (300mgI/ml), with the dosage of 150-250 ml. The time window for arterial thrombolysis (from the initial onset to the onset of arterial thrombolysis) is 3-6 hours. Thrombolysis lasts for 30 minutes to 2.5 hours. The thrombolytic agent used was urokinase. Doses of urokinase ranged from 60000 to 600000 U, with 10 mL saline/60000 U, in boluses. 40 of the patients were treated with thrombolysis alone and 57 were treated with mechanical thrombectomy combined with arterial thrombolysis. Among the 97 patients, the site of occlusion was the internal carotid artery in 32 patients, the M1 segment of middle cerebral artery in 54 patients, the M2 segment in 8 patients, and the basilar artery in 3 patients.

### 2.3. CT Acquisition

After cerebral angiography and revascularization of obstructed vessels, all patients underwent non-enhanced CT scan of brain immediately after AR. Follow-up CT was performed within 24 hours or 48 hours after the procedure. Gd-free MR scanning was performed in 21 patients within 48 hours after procedure. Using Philips Brilliance 256 rows of iCT scanners, all patients were scanned from the base of the skull to the top of the skull. Scanning conditions: 120KV, 300MA, layer thickness of 3 mm. Philips Achieva 1.5 T MR scanner was used to collect the images with the skull phased-front circle. The scanning sequence includes T1-weighted sequence, T2- weighted sequence, fluid attenuated inversion recovery (Flair), diffusion weighted imaging (DWI), apparent diffusion coefficient (ADC), susceptibility weighted imaging (SWI) etc.

### 2.4. Imaging Evaluation

The characteristics of non-enhanced brain CT of all patients were analyzed and evaluated by two experienced attending radiologists or above. According to the shape, location and with/without mass effect of hyperdense lesions, the patients were divided into three categories: type I (sporadic patchy lesions with unclear boundaries which mostly distributed in the cerebral cortex and sulti, without mass effect (Figure 1(a))), type II (solid “mass” shaped lesions with well-defined boundaries which mostly distributed in the basal ganglion and without mass effect or mild mass effect (Figures 2(a) and 3(a))) and type III (diffuse patchy lesions occupying a larger area with obvious mass effect (Figure 4(a))). Once divergence occurred during the diagnosis and classification evaluation, the two parties shall solve the difference through consultation.

### 2.5. Statistical Analysis

All statistical analyses were conducted using SPSS version 18 (SPSS Inc, Chicago, USA). Quantitative data were expressed as means ± standard (SD) and compared by the two-sample independent Student's t-test; Qualitative data was expressed as rate and compared by Chi-square test. P < 0.05 indicated that the difference was statistically significant.

## 3. Results

### 3.1. Overall Results

Among 97 patients, 52 (53.6%) patients showed hyperdense lesions around the intracranial infarction area on non-enhanced CT conducted immediately after AR, whereas the other 45 (46.4%) patients (the control group) had no hyperdense lesions. The basic clinical data of patients in the hyperdense group and without hyperdense group were summarized in Table 1. There were no significant differences in age, sex, hypertension, diabetes, NIHSS score, history of antiplatelet therapy before onset, degree of recanalization, methods of arterial revascularization. 30 (57.7%) patients in the intracranial hyperdense lesions group developed HT after AR, Among the control group, 7 patients converted to AICH (Asymptomatic Intracranial Hemorrhage) in follow-up CT/MR within 24 or 48 hours after AR (Table 2), and no SICH occurred. Significantly higher HT incidence was observed in the hyperdense lesions group when compared with the without hyperdense lesions group (P < 0.001).

### 3.2. Outcome of the Hyperdense Lesions

In the hyperdense group, hyperdense lesions were completely disappeared in 22 (42.3%) patients (Figures 1 and 3), 23 (44.2%) patients displayed contrast extravasation combined with HT (Figure 2) and 7 (13.5%) patients were confirmed SICH (Figure 4) in follow-up CT/MR within 24 or 48 hours after AR. In follow-up CT 24 or 48 hours after AR, the outcome of different types of hyperdense lesions were as follows (Table 3): sporadic patchy type I lesions (16 lesions) were completely disappeared, showing contrast extravasation; 23 type II lesions (74.2%) turned to hemorrhage (AICH), 2 lesions (6.5%) revealed SICH and 6 lesions (19.4%) were contrast extravasation; all of the type III (5 cases) lesions developed into SICH. Type II and type III had a significantly higher incidence of HT than type I (P < 0.01). The sensitivity, specificity, positive predictive value and negative predictive value of hyperdense lesions on non-enhanced CT conducted immediately after AR for the prediction of HT were 81.1%, 63.3%, 57.7% and 84.4%, respectively.

## 4. Discussion

With the development of medical imaging equipment and interventional medical technology, patients with AIS have more opportunities for transductal AR (including intra-arterial drug thrombolysis, mechanical thrombectomy), which improves the rate of vascular recanalization in stroke patients and greatly improves the patients' clinical prognosis and survival rate. However, intracranial hemorrhage, a complication associated with intravascular interventional procedures, poses a challenge to clinical diagnosis and treatment of AIS. Immediately after completing intra-arterial procedures, a non-enhanced CT is often performed to assess the progression of the AIS and whether hemorrhage has occurred [6]. Non-enhanced CT often detects hyperdense lesions in the parenchyma. Not all hyperdense lesions on non-enhanced CT conducted immediately after AR represent hemorrhage, it may be attributed to either contrast extravasation or cerebral hemorrhage [6, 8]. So neurologists and neuroradiologists need to identify the true nature of the hyperdense lesions so that appropriate interventions can be taken in time, otherwise it will seriously affect the prognosis of patients.

A large amount of contrast agent is injected during the angiography and AR in patients with AIS, so extravascular exudation of contrast agent may be the pathological mechanism of CT intracranial hyperdense lesions. Contrast extravascular exudation is based on damage to the blood-brain barrier (BBB) [9]. For patients with AIS, the permeability of occluded vessels in the infarcted area was changed. After recanalization, the blood flow in the infracted area increased significantly and hyperperfusion occurred. When the perfusion pressure of the distal capillary bed exceeds the bearing capacity of the vessel wall, the BBB is destroyed and contrast agent exudates. The removal time of the contrast agent injected during the recanalization is prolonged due to ischemia and hypoxia in the cerebral infarction area, which results in the local retention of contrast agent [10]. During interventional procedure, microcatheter and microguide wire may lead to vascular intimal damage, which is also one of the common causes of contrast extravasation [11, 12]. The manifestations of post-procedure CT intracranial hyperdense lesions vary with the degree of cerebral microvascular injury. When ischemic injury only destroys the permeability barrier of endothelial cells, the intracranial hyperdense lesions may be a single contrast agent without hemorrhage. However, when ischemic infarcts break down the structural barrier-basement membrane, the hyperdense lesions may be associated with some form of hemorrhage, or a mixture of contrast and blood. Disruption of the blood–brain barrier may be an essential condition for hemorrhagic transformation [11–13].

There were no significant differences in terms of age, sex, hypertension, diabetes mellitus, National Institute of Health Stroke Scale score (NIHSSs), history of antiplatelet therapy before onset, recanalization rate and method of thrombolysis between patients with intracranial hyperdense lesions group and those without. The incidence of HT in patients with hyperdense lesions group was significantly higher than that without hyperdense lesions group, and the difference was statistically significant (Table 1).

In this study, 22 (42.3%) patients of the intracranial hyperdense lesions were completely disappeared on a follow-up CT obtained within 24 hours or 48 hours after procedure. Among them, 16 patients had type I hyperdense lesions and 6 patients had type II lesions. Follow-up CT scan showed no recurrence of HT in these patients. This rapidly fading intracranial hyperdense lesions was contrast extravasation without HT. That is, ischemic injury in these patients may be limited only to the endothelial permeability barrier. Wildenhain et al. reported that rapid dissolution of intracranial hyperdense lesions is a good prognostic indicator [2].

There are several definitions of contrast extravasation after AR in patients with AIS. Nakano et al. [14] believed that the rapidly fading of high-density shadow was the main basis for the diagnosis of the extravasation of contrast agent. Mericle et al. [7] showed that extravasation of contrast medium should be defined as a hyperdense lesions with a maximal Hu measurement>90 and/or the hyperdense lesions rapidly subsided within 24 hours after AR. According to our study, we are more inclined to suggest that rapid resolution of intracranial hyperdense lesions is the key to the diagnosis of contrast extravasation, and there was no mass effect of the intracranial hyperdense lesions. The maximal Hu measurement>90 of intracranial hyperdense lesions was not an absolute indication for the diagnosis of the extravasation of contrast medium.

If follow-up CT within 24 hours or 48 hours after procedure showed that the attenuation of the intracranial hyperdense lesions was mildly reduced compared with that of non-enhanced CT conducted immediately after completing inter-arterial procedure, and the size and contour of intracranial hyperdense lesions changed slightly, even the hyperdense lesions appeared space occupying effect. The above CT findings are known as contrast extravasation combined with HT. HT is the most serious complication after AR in AIS patients [12]. HT after arterial thrombolysis can be divided into SICH and AICH. SICH was defined as a decrease in the NIHSSs ≥4 within 36 hours after thrombolysis and intracranial hemorrhage confirmed by imaging was correlated with the deterioration of clinical symptoms in time. AICH was defined as bleeding without deterioration of neurological symptoms [15].

HT is a complex and multifactorial phenomenon. Known risk factors include age, blood glucose, low platelet count, high NIHSSs, size and location of ischemic area, poor collateral vessels, arterial stiffness, thrombolytic agent used and time window allowed for the initiation of the therapy [16, 17]. And its occurrence is closely related to the damage of BBB, the reperfusion injury of ischemic area, the use of microcatheter, the establishment of collateral circulation and prolonged procedure time [18, 19], which is the result of the combined action of the above factors [4]. In this study, 30 (57.7%) patients in the intracranial hyperdense lesions group developed HT after AR, including 23 (44.2%) patients with AICH and 7(13.5%) patients with SICH. All of the 23 (44.2%) patients with AICH were type II hyperdense lesions. Among the 7 patients with SICH, 2 were type II hyperdense lesions and 5 were type III.

SICH, a massive intracerebral hematoma (accompanied by obvious space occupying effect) with worsening neurological symptoms, is a clinical and CT imaging hybrid [20]. It is also the most intractable problem in the reperfusion treatment of AIS patients. The rapid disappearance of intracranial hyperdense lesions after AR had nothing to do with SICH. Since SICH is a serious microvascular injury involving the basement membrane, no hyperdense lesions on non-enhanced CT immediately after AR suggests that the permeability and structural barrier of microvascular endothelial cells are not destroyed, which may be a reliable negative predictor of SICH, in other words, the incidence of SICH will be extremely low or will not occur at all. Kass-Hout et al. [21] indicated that a longer procedure time is an independent predictor for SICH in patients receiving mechanical thrombectomy. The extended procedure time may be due to difficulty getting catheters into blocked vessels, which may be related to arterial stiffness or more comorbidities [22]. Prolonged procedure time means more attempts to recanalize the occluded vessels. The above factors could greatly increase the incidence of HT [23, 24]. A prolonged procedure time was significantly associated with a higher rate of SICH, even in patients with successful recanalization [19].

Nakano et al. [14] reported that 48% of patients showed intracranial hyperdense lesions on non-enhanced CT immediately after arterial thrombolysis, and 29.7% of these patients developed SICH, while patients without intracranial hyperdense lesions on non-enhanced CT immediately after AR had no SICH. Jang et al. [6] reported that 33% (31/94) of patients displayed intracranial hyperdense lesions on non-enhanced CT immediately after intraarterial procedures. Among them, 58% (18/31) developed cerebral hemorrhage, and 19.4% (6/31) developed SICH. In this study, 53.6% (52/97) of the patients showed intracranial hyperdense lesions around the intracranial infarction area on non-enhanced CT immediately after AR, and 13.5% (7/52) of them developed SICH. None of the patients without intracranial hyperdense lesions developed SICH. In our study, the incidence of intracranial hyperdense lesions on non-enhanced CT immediately after AR was higher than that in the results of Nakano et al. [14] and Jang et al. [6], and the incidence of SICH was lower than that in the results of Nakano et al. [14] and Jang et al. [6]. There was no significant difference between cases selection and vascular reconstruction methods, so this difference may be related to the insufficient sample size, different generations of thrombectomy devices and procedure time. Whether it is related to other factors remains further analysis with a larger group of patients. Our results showed that none of the patients without intracranial hyperdense lesions developed SICH, which was consistent with the study of Nakano et al. [14].

This study showed that type I intracranial hyperdense lesions (sporadic patchy lesions with unclear boundaries), which completely disappeared within 24 hours post-procedure, is a single, pure contrast extravasation. A large proportion (80.6%,25/31) of type II intracranial hyperdense lesions (solid “mass” shaped lesions with well-defined boundaries) converted to hemorrhage, while a small proportion (19.4%,6/31) were only contrast extravasation. Type III intracranial hyperdense lesions (diffuse patchy lesions with mass effect) invariably developed into SICH. The occurrence of intracranial hyperdense lesions after AR has a high sensitivity and negative predictive value for the prediction of cerebral HT, but the specificity and positive predictive value are not high, which is consistent with the research results of Kim et al. [25].

This study has some limitations. Firstly, the retrospective design has its inherent limitations of such study. Secondly, the sample was small, which may have influenced the results in this study. Another limitation is that our study was a single-center study and we did not analyze the effect of the duration of procedure on the occurrence of hyperdense lesions on non-enhanced CT conducted immediately after AR. Therefore, we will conduct multicenter studies in future to collect more cases of ischemic stroke with transarterial revascularization and follow up for a longer time, so as to confirm the availability and practicability of the morphological classification of intracranial hyperdense lesions in the current study.

## 5. Conclusions

In conclusion, the occurrence of intracranial hyperdense lesions on non-enhanced CT conducted immediately after AR has its limitations for the accurate prediction of cerebral HT (including SICH and AICH). Type I hyperdense lesions suggested pure contrast extravasation and was not associated with hemorrhagic complications. The presence of Type II and type III hyperdense lesions indicated higher incidence of HT, in particular, the presence of type III hyperdense lesions indicated an ominous outcome. When intracranial hyperdense lesions of type II and type III appear around the intracranial infarction area in stroke patients, high attention should be paid to the progress of the patient's neurological symptoms and timely and effective treatment should be given to minimize the complications of cerebral hemorrhage.

## Figures and Tables

**Figure 1:** Non-enhanced brain CT scan of a 58-year-old woman who had a sudden onset of impaired left limb movement. (a). The non-enhanced brain CT scan obtained immediately after intra-arterial thrombolysis showed that a type I hyperdense lesion was located in the right temporal lobe cortex with a CT value of 90-135 Hu. There was no mass effect. (b). Follow-up CT scan obtained 24 hours after the end of AR, the hyperdense lesion on the right temporal lobe cortex was completely disappeared.

**Figure 2:** CT scan of a 62-year-old man who had a sudden onset of impaired right limb movement. (a). The non-enhanced brain CT scan obtained immediately after intra-arterial thrombolysis showing a hyperdense area in the head portion of the left caudate nucleus and the entire left lentiform nucleus. Representative type II, namely solid “mass” shaped lesions with well-defined boundaries and without mass effect. (b). Follow-up CT scan obtained 48 hours after the end of intra-arterial thrombolysis. The range of the hyperdense area increased slightly and the attenuation decreased. The patient was not accompanied by deterioration of neurological symptoms. (c). On the 2nd day after the procedure, susceptibility weighted imaging showed patchy low signal in the left basal ganglia region, indicating hematoma formation. (d). Two weeks after the procedure, the left basal ganglia hematoma had been completely absorbed.

**Figure 3:** CT scan of a 58-year-old woman who had a sudden onset of impaired left limb movement. (a). The non-enhanced brain CT scan obtained immediately after intra-arterial thrombolysis showing a type II hyperdense lesion in the right lentiform nucleus with a CT value of 90-135 Hu. A type I hyperdense lesion was located in the right insular cortex with a CT value of 52-57 Hu (the latter was not included in this study). There was no mass effect in the above two lesions. (b). Follow-up CT scan obtained 24 hours after the end of AR, the hyperdense lesion of the right lentiform nucleus was obviously absorbed. The patient was not accompanied by deterioration of neurological symptoms.

**Figure 4:** CT scan of a 66-year-old woman who experienced a sudden left limb inactivity accompanied by loss of speech function for 4 hours. There was no intracranial hemorrhage on CT scan before thrombolytic therapy. (a). The non-enhanced brain CT scan obtained immediately after intra-arterial thrombolysis showing a type III hyperdense lesion in the right basal ganglia with a CT value of 55-73 Hu. The right ventricle was significantly compressed. The patient had a marked symptom of neurological deterioration. (b). Follow-up CT scan obtained 24 hours after the end of AR revealed that the contour of the hyperdense lesion located in the right basal ganglia region was slightly expanded, the attenuation was increased, and the surrounding low-density edema occurred, with obvious space-occupying effect. (c). T2WI and D FLAIR obtained 24 hours after procedure showed large patchy low signals in the right basal ganglia region surrounded by high signal. Low signal denotes hematoma and high signal denotes edema.

**Table 1:** Baseline Characteristics of Patients in the Hyperdense Group and without hyperdense Group.

	Hyperdense group (n = 52)	Without hyperdense group (n = 45)	P
Age (mean ± SD)	61.5 ± 8.66	62.0 ± 8.26	0.773
Gender (male/female)	28/24	23/22	0.788
Hypertension	24	20	0.866
Diabetes	18	14	0.714
NIHSS score (mean ± SD)	13.94 ± 3.9	13.93 ± 4.2	0.991
History of antiplatelet therapy before onset	29	25	0.983
Successful recanalization (%)	34 (65.4)	26 (57.8)	0.442
Thrombolysis	22	18	0.818
Thrombolysis and mechanical thrombectomy	30	27	0.818
HT (%)	30 (57.7)	7 (15.6)	<0.001

NIHSS=National Institute of Health Stroke Scale. HT = hemorrhagic transformation.

**Table 2:** Distribution of HT between the hyperdense group and the without hyperdense group.

	No hemorrhage	AICH	SICH
Hyperdense group (n = 52)	22	23	7
Without hyperdense group (n = 45)	38	7	0
P		<0.001	

HT = hemorrhagic transformation, AICH = Asymptomatic Intracranial Hemorrhage, SICH = Symptomatic Intracranial Hemorrhage.

**Table 3:** Distribution of HT among the different types of hyperdense lesions.

	No hemorrhage	AICH	SICH
Type I (n = 16)	16	0	0
Type II (n = 31)	6	23	2
Type III (n = 5)	0	0	5
P		<0.01	

HT = hemorrhagic transformation, AICH = Asymptomatic Intracranial Hemorrhage, SICH = Symptomatic Intracranial Hemorrhage.

## Data Availability

The data used to support the findings of this study are included within the article.
